# Somatic ‘Soluble’ Adenylyl Cyclase Isoforms Are Unaffected in Sacy^tm1Lex^/Sacy^tm1Lex^ ‘Knockout’ Mice

**DOI:** 10.1371/journal.pone.0003251

**Published:** 2008-09-22

**Authors:** Jeanne Farrell, Lavoisier Ramos, Martin Tresguerres, Margarita Kamenetsky, Lonny R. Levin, Jochen Buck

**Affiliations:** Department of Pharmacology, Weill Medical College of Cornell University, New York, New York, United States of America; Texas Tech University Health Sciences Center, United States of America

## Abstract

**Background:**

Mammalian Soluble adenylyl cyclase (sAC, Adcy10, or Sacy) represents a source of the second messenger cAMP distinct from the widely studied, G protein-regulated transmembrane adenylyl cyclases. Genetic deletion of the second through fourth coding exons in Sacy^tm1Lex^/Sacy^tm1Lex^ knockout mice results in a male sterile phenotype. The absence of any major somatic phenotype is inconsistent with the variety of somatic functions identified for sAC using pharmacological inhibitors and RNA interference.

**Principal Findings:**

We now use immunological and molecular biological methods to demonstrate that somatic tissues express a previously unknown isoform of sAC, which utilizes a unique start site, and which ‘escapes’ the design of the Sacy^tm1Lex^ knockout allele.

**Conclusions/Significance:**

These studies reveal increased complexity at the sAC locus, and they suggest that the known isoforms of sAC play a unique function in male germ cells.

## Introduction

In mammals, the widely studied second messenger cAMP can be generated by two types of enzymes: G protein-regulated transmembrane adenylyl cyclases (tmACs) and bicarbonate-regulated soluble adenylyl cyclase (sAC). Nine distinct genes encode a family of tmAC isoforms which display differential tissue distribution and responsiveness to calcium. Each tmAC isoform is modulated by heterotrimeric G proteins in response to hormones and neurotransmitters (reviewed in [1]). In contrast, a single sAC gene [2] generates multiple isoforms by alternative splicing [3], [4] whose activities are directly stimulated by bicarbonate and calcium ions [5]–[8]. A second sAC-related locus present in human, dog and other mammalian genomes, but not detected in mouse or rat genomes, appears to be a pseudogene [9].

The sAC protein was initially purified from rat testis cytosol, and two independent cDNAs, which were subsequently shown to represent alternatively spliced isoforms [4], were cloned from a rat testis cDNA library [2]. These two transcripts were termed full-length (sAC_fl_), encoding a 187 kD protein, and truncated (sAC_t_), encoding a 53 kD protein (Fig. 1A). The protein originally purified corresponds to sAC_t_. This isoform is highly active but of relatively low abundance. We required approximately 1000 rat testis to recover sufficient material to obtain sequence information [2], [10], and detecting sAC_t_ in testis cytosol from wild type mice by Western blotting required an initial enrichment step; i.e., immunoprecipitation with a different sAC-specific monoclonal antibody [11]. The majority of immune reagents generated, protein biochemistry and kinetics, and the design of a knockout mouse have been based on the knowledge of the sAC_t_ and sAC_fl_ isoforms.

**Figure 1:** Schematic organization of (A) previously identified, testicular sAC transcripts and (B) the newly identified somatic sAC transcript. Boxes denote exons. C1 and C2 refer to the two catalytic domains. Red exons contain stop codons. (A) sAC_fl_ is encoded by all known coding exons (32), and sAC_t_ is generated by skipping exon 12. Yellow exons (2-4) are removed in the Sacy^tm1Lex^ allele. Arrows indicate approximate locations of epitopes for the indicated monoclonal antibodies (R40, R21, and R37). (B) Somatic sAC transcripts derive from a unique start site upstream of exon 5 and continue through at least exon 16 to an unknown stop.

Historically, ‘soluble’ adenylyl cyclase activity had only been detected in testis cytosol [12], [13]. Initial Northern blot data confirmed that sAC message is abundant in testis [2], and that it is specifically enriched within the developing male germ cells [14]. But more sensitive methods of mRNA detection, including RT-PCR [14] and multiple tissue expression arrays [15], revealed sAC mRNA to be universally expressed. For example, the NCBI Gene Expression Omnibus database chronicles sAC expression in a number of somatic tissues, including brain. Finally, the GNF gene expression Atlas and in situ analysis performed by the Allen Brain Institute identified sAC message throughout the nervous system including dorsal root ganglia, spinal cord, cerebellum, hypothalamus, and thalamus [16].

To examine sAC protein expression, we and others, have raised various polyclonal antisera and numerous monoclonal antibodies against sAC [3], [4], [6], [17], [18]. These immune reagents predict sAC to also be expressed in a large number of cell lines [3], [18] and a variety of somatic tissues [6], [17], [19]–[24] However, the sAC protein identified in cells and tissues tends to be associated with intracellular organelles [18], [24], [25] or vesicles [20], implying that somatic sAC is not a soluble protein but could require detergent extraction.

Somatic functions for sAC are predicted by both genetic and pharmacologic experiments. The human sAC locus was implicated in familial absorptive hypercalciuria (AH) [15], a syndrome of calcium homeostasis defects in intestine, kidney and bone. Pharmacological methods taking advantage of sAC-selective versus tmAC-selective inhibitors have identified a role for sAC as a cellular sensor of pH_i_ in epididymis [19] and kidney [20], a CO_2_/HCO_3_ sensor in airway cilia [21], a mediator of oxidative burst in response to tumor necrosis factor in human neutrophils [26], and a modulator of the Cystic Fibrosis Transmembrane Conductance Regulator (CFTR) in corneal endothelium [22] and in human airway epithelium [17]. In certain isolated primary cells and cell lines, we have been able to use sAC-specific RNAi mediated knockdown to confirm results obtained with sAC- and tmAC-selective pharmacological inhibitors. Using these more stringent criteria, we have elucidated additional roles for sAC in neuronal responses to the guidance cue Netrin-1 [23] and in cellular responses to the neurotrophin, Nerve Growth Factor (NGF) [27], [28].

These numerous putative somatic functions for sAC are inconsistent with the initial descriptions of a very specific germ cell phenotype in the existing sAC knockout (Sacy^tm1Lex^/Sacy^tm1Lex^) mouse [11], 29, 30. These mice were generated by homologous recombination with an exon trapping, IRES-lacZ expression cassette replacing the 2^nd^ through 4^th^ coding sequence exons present in both sAC_t_ and sAC_fl_ isoforms [29]. In mice with the Sacy^tm1Lex^ locus, lacZ expression was only detected in testis, suggesting that at least the promoter and exon 1 are specific to male germ cells. More importantly, homozygous male knockout mice are sterile; their sperm are immotile, do not undergo capacitation, and are unable to fertilize an egg *in vitro* [11], [29]. A more extensive phenotypic analysis revealed that female Sacy^tm1Lex^/Sacy^tm1Lex^ mice display increased circulating cholesterol and triglyceride levels and both male and female homozygous knockout animals have slightly elevated heart rates [as deposited in the Mouse Genome Database [31]]. And even though knockout phenotypes are often muted or absent due to compensation, such subtle somatic phenotypes are unexpected considering the variety of physiological functions demonstrated or predicted for sAC. For example, even though we demonstrated that sAC is essential for Netrin-1 induced axonal outgrowth in commissural axons [23], Sacy^tm1Lex^/Sacy^tm1Lex^ mice do not exhibit the pronounced structural brain defects [23], [30] seen in Netrin-1 knockout animals [32].

Moe and co-workers cloned human sAC cDNAs from somatic cells whose open reading frames do not contain exons deleted in Sacy^tm1Lex^/Sacy^tm1Lex^ mice [3]. If such cDNAs represent the predominant species of sAC in mammalian somatic tissues, it would explain how the Sacy^tm1Lex^ knockout could exhibit exclusively a germ cell phenotype. Here we use immunological and molecular methods to confirm the existence of previously unknown somatic isoforms of sAC. These somatic sAC isoforms derive from a unique mRNA start site which “escapes” the design of the Sacy^tm1Lex^ mouse.

## Results

### sAC-specific antibodies identify isoforms unaffected in Sacy^tm1Lex^ ‘knockout’

We used two sAC-specific monoclonal antibodies recognizing distinct, non-overlapping epitopes to examine the molecular nature of sAC proteins expressed in brain. R21 is a monoclonal antibody recognizing an epitope in coding sequence exon 5 (within amino acids 206–216) of sAC_fl_ while R37 is a monoclonal antibody recognizing an epitope in exon 11 (within amino acids 436–466) (Fig. 1). Due to compelling evidence for a function of sAC in neuronal signaling [23], [27] and because we previously demonstrated we could recover sAC activity (i.e., it was inhibited by the sAC-specific inhibitor, KH7, and it was insensitive to the tmAC activator, forskolin) by R37 immunoaffinity purification from detergent extracts of rat brain [23], we first focused on the sAC proteins present in mouse brain. Western blots using R21 revealed a number of immunoreactive bands. Surprisingly, none of these putative sAC bands were altered in the Sacy^tm1Lex^/Sacy^tm1Lex^ mice (Fig. 2A, first two lanes).

**Figure 2:** Somatic sAC isoforms unaffected in Sacy^tm1Lex^ locus. Immunoprecipitations (IP) using mAb R37 or IgG control antibody from detergent solubilized whole cell extracts (lysates) of brains (A,B) or kidney (C) from wild type or Sacy^tm1Lex^/Sacy^tm1Lex^ mice were subjected to Western analysis using (A,C) biotinylated R21 mAb (R21B) or (B) biotinylated R37 mAb (R37B). White circles denote nonspecific bands detected with streptavidin (no primary antibody) alone. The smear at ∼50 kDa in the R37 IP from brain resolves to at least two bands when less of the IP is loaded for Western blotting (inset).

We also examined the sAC activity immunoprecipitated by R37 from wild type and Sacy^tm1Lex^/Sacy^tm1Lex^ brains (Fig 3). We previously showed the adenylyl cyclase activity immunoaffinity purified from wild type mouse brains was insensitive to forskolin and inhibited by sAC-specific inhibitor [23]. Preliminary analysis suggests that there is considerably less sAC adenylyl cyclase activity immunoprecipitated from a single wild type brain (77 pmol cAMP/ml) than from wild type testis (at least 254 pmol cAMP/ml) (Fig. 3A). This is not surprising considering sAC mRNA expression in testis is greater than in any somatic tissue, including brain [14], and because testis expresses the highly active, sAC_t_ isoform [5], [11]. Equivalent amounts of adenylyl cyclase activity were immunoprecipitated from wild type or Sacy^tm1Lex^/Sacy^tm1Lex^ brains (Fig. 3B), and the activity from Sacy^tm1Lex^/Sacy^tm1Lex^ brains was confirmed to be sAC by its insensitivity to forskolin (no statistically significant difference in the presence or absence of 10 μM forskolin) and its sensitivity to the sAC-selective inhibitor, 4-hydroxyestradiol. The sAC-selective catechol estrogen, 4-hydroxyestradiol [19], [33], [34], was used to inhibit the immunoprecipitated activity from Sacy^tm1Lex^/Sacy^tm1Lex^ brains because it is unaffected by the detergents used during immunoprecipitation. The immunoprecipitated activity from Sacy^tm1Lex^/Sacy^tm1Lex^ brains was inhibited by approximately 50% in the presence of catechol estrogen (Table 1). These data suggested that the sAC protein(s) in brain was unaffected by the deletion of exons 2-4, and would therefore represent novel, previously uncharacterized isoforms.

**Figure 3:** Somatic sAC activity in brain is lower than activity in testis, but it is not diminished in brains from Sacy^tm1Lex^/Sacy^tm1Lex^ mice. (A) Adenylyl cyclase activity (in pmol cAMP formed per ml) in mouse IgG or R37 IP from detergent extracts from a single mouse brain or mouse testis from wild type mice. Activity from testis may be under-represented; we did not confirm antibody was in excess. MM is adenylyl cyclase reaction conditions alone (no IP added). Control IgG activity is derived from pooled brain and testis detergent extracts. Values represent averages of duplicate determinations. (B) Adenylyl cyclase activity in R37 IPs from wild type (WT) or Sacy^tm1Lex^/Sacy^tm1Lex^ (KO) mice. MM is adenylyl cyclase reaction conditions alone (no IP added). Extracts were precleared through mouse IgG prior to immunoprecipitation. Values represent quadruplicate determinations from two wild type and two knockout brains with error bars indicating S.E.M.

**Table 1:** sAC activity from Sacy^tm1Lex^/Sacy^tm1Lex^ brains

	cAMP* (pmol/mL)	Standard Deviation (pmol/mL)
Basal activity	20.472	4.138
4-hydroxyestradiol (100 μM)	11.223	0.726

* Average of quadruplicate determinations.

To determine whether the immunoreactive bands were recognized by both antibodies, which would provide a compelling argument that they are *bona fide* sAC isoforms, we immunoprecipitated using R37 followed by Western blotting with R21 (biotinylated R21 was used for Western blotting to prevent detection of the immunoprecipitating R37 IgG). Western blotting the R37 immunoprecipitates reveals that at least two of the immunoreactive bands, at approximately 50 kDa, are recognized by both sAC-specific monoclonal antibodies (Fig. 2A,B). These two proteins are also diminished in the brain extracts following specific (R37) immunoprecipitation, but remain in brain extracts following immunoprecipitation with control (isotype-matched IgG) antibody. Thus, we have identified two proteins of approximately 50 kDa proteins, which are recognized by distinct sAC-specific monoclonal antibodies and are correlated with sAC-like adenylyl cyclase activity. Yet, both isoforms are unaffected in brains from Sacy^tm1Lex^/Sacy^tm1Lex^ mice.

If these brain sAC isoforms were unaffected by removal of exons 2-4, they should not be recognized by antisera directed against this region. One of our monoclonal antibodies, R40, recognizes an epitope which spans exons 2 and 3 (Fig. 1A). Using R40, we were able to immunoprecipitate a 50 kDa protein from wild type mouse testis cytosol, which was absent in testis cytosol from Sacy^tm1Lex^/Sacy^tm1Lex^ mice (Fig. 4, top). This 50 kDa isoform is presumably sAC_t_. Not only was this isoform not detectable in brain, but this exon 2-3 directed monoclonal antibody did not immunoprecipitate any detectable sAC isoforms from wild type or Sacy^tm1Lex^/Sacy^tm1Lex^ brains (Fig. 4, bottom). The testis cytosolic isoform, sAC_t_, and one of the newly identified detergent extractable, brain isoforms run together at ∼50 kDa and are not easily distinguished on SDS/PAGE (compare Fig. 2 and 4). We believe this coincidence has contributed to previous confusion about the molecular identity of sAC isoforms identified by Western blotting.

**Figure 4:** Sperm sAC isoforms are not detected in brain. Immunoprecipitations (IP) using mAb R40 or isotype-matched IgG control antibody from detergent solubilized whole cell extracts (lysates) of testis (top) or brain (bottom) from wild type or Sacy^tm1Lex^/Sacy^tm1Lex^ mice were subjected to Western analysis using biotinylated R21 mAb. The sharp band at ∼50 kDa in the R40 IP from wild type testis is distinct from the faint, background bands found in Sacy^tm1Lex^/Sacy^tm1Lex^ mice and in the control IgG IP.

We next asked whether the detergent extractable, 50 kDa isoforms present in brain could be found in other somatic tissues. In kidney, sAC has been proposed to form a complex with the vacuolar proton ATPase to regulate renal distal proton secretion [20]. Western blots (using R21) of R37 immunoprecipitates from detergent extracts of wild type and Sacy^tm1Lex^/Sacy^tm1Lex^ kidneys revealed a ∼50 kDa sAC isoform, which once again, was unaffected by removal of exons 2-4 (Fig. 2C). These data suggest that at least one of the two ∼50 kDa brain isoforms represents a widely distributed, somatic isoform of sAC.

### sAC transcripts in brain use an alternate start site

We used the knowledge that brain sAC isoforms must contain the epitopes recognized by R21 (amino acids 206–216) and R37 (amino acids 436–466) to explore the nature of brain sAC cDNAs. Using primers specifically recognizing these sequences and 35 cycles of amplification, we detected a fragment in brain mRNA from wild-type mice; with forty rounds of amplification, we amplified fragments from both wild type and Sacy^tm1Lex^/Sacy^tm1Lex^ brains (Fig. 5). In each case, nucleotide sequencing confirmed the amplified fragment contained a single product corresponding to the complete sequence (i.e., contained all known exons) between exons 5 and 11. The need for greater than 30 rounds of amplification to detect sAC message in somatic tissues is consistent with the recently published identification of sAC mRNAs in specific neuronal cell types [30]. PCR amplification of the LacZ/Neo cassette confirmed the identity of Sacy^tm1Lex^/Sacy^tm1Lex^ tissues, but it is unclear why knockout brains and testis appear to express equivalent LacZ/Neo message.

**Figure 5:** RT-PCR of cDNA from testis and brain from wild type (WT) and Sacy^tm1Lex^/Sacy^tm1Lex^ mice (KO). (A) PCR across exons 15-16. (B) PCR across exons 5-11. (C) PCR for β-actin loading control. (D) PCR for LacZ/Neo. (−) is a no template control. The number in the lower right corner of each panel is the number of cycles used in each experiment.

Consistent with the facts that R40 did not detect any sAC isoforms in brain and the isoforms we do detect in brain are unaffected by removal of exons 2-4, we were unable to amplify a product using exon 1, 2, 3, or 4 sense primers to exon 5 antisense primers from either wild type or knockout brain mRNA (Fig. 6 and data not shown). As control, the exon 1 sense and exon 5 antisense primers amplified the expected size product using testis mRNA from wild type and Sacy^tm1Lex^/+ heterozygous mice (Fig. 6). These primers also amplified a smaller product (of 200 base pairs) from Sacy^tm1Lex^/+ heterozygous and Sacy^tm1Lex^/Sacy^tm1Lex^ homozygous knockout mice which nucleotide sequencing confirmed to be an in-frame, exon1:exon5 spliced product arising exclusively from the Sacy^tm1Lex^ allele. It is possible this uniquely spliced product in testis from knockout mice is responsible for the residual adenylyl cyclase activity identified in sperm from Sacy^tm1Lex^/Sacy^tm1Lex^ mice [35]. It is also possible this aberrant, testis-specific product diminishes splicing into the LacZ/Neo cassette, explaining why the level of LacZ/Neo message in testis is not much higher than the levels found in brain (Fig. 5).

**Figure 6:** PCR from Exons 1 through 5 from WT and knockout mouse tissues. (A) and (C) PCR across exons 1-5. (A) Testis first strand from WT (+/+), Sacy^tm1Lex^/+ heterozygote (+/−), and Sacy^tm1Lex^/Sacy^tm1Lex^ homozygous knockout (−/−) mice. (C) First strand cDNA from brain (B), heart (H), kidney (K), or liver (Li) from Sacy^tm1Lex^/Sacy^tm1Lex^ homozygous knockout (−/−) mice; (−) indicates no template control. (B) and (D) β-actin controls. The number in the lower right corner of each panel is the number of cycles used in each experiment.

To test whether brain sAC mRNAs use an alternate start site, we performed 5′ Rapid Amplification of cDNA Ends (RACE) starting in exon 5. We obtained two 5′ RACE products, which extended beyond the intron/exon boundary of exon 5 into the sequence previously thought to be intron. The two fragments were contiguous; the larger fragment simply extended further (344 nucleotides) into the intron upstream of coding exon 5 (Fig. 7; GenBank Accession #EU478437). Neither fragment extended into sequences removed in the Sacy^tm1Lex^ locus, and these upstream sequences did not correspond to any of the alternatively spliced transcripts identified in human tissues [3]. Thus, sAC mRNAs in mouse brain appear to utilize a unique start site, which would not be deleted in Sacy^tm1Lex^/Sacy^tm1Lex^ mice (Fig. 1B).

**Figure 7:** Sequence of 5′ RACE product defining new mRNA start site from mouse brain. Sequence in bold is the newly defined 5′UTR which corresponds to the region previously assigned to be the intron between Exons 4 and 5.

We had first concluded that sAC is widely distributed in mammals based upon an RT-PCR experiment using primers in exons 15 and 16 [14]. Reed *et al*. reached a similar conclusion using an overlapping region as probe in a multiple tissue array blot [15]; therefore, exon 16 is likely included in somatic isoforms of sAC. Using a sense primer corresponding to the newly identified 5′ end and an antisense primer in exon 16, we amplified a single product, from both wild type and Sacy^tm1Lex^/Sacy^tm1Lex^ mouse brain mRNA, which extended from the newly described start site through exons 5 to 16 (Fig. 1B). This cDNA was amplified in both wild type and Sacy^tm1Lex^/Sacy^tm1Lex^ brains. While we still do not know the true 3′ end of brain sAC cDNAs, we expect them to be significantly shorter than sAC_fl_ because the encoded protein isoforms are only ∼50 kDa. Consistent with this, we were unable to amplify a product from the new start site to exon 32 (data not shown). This new mRNA start site, outside the region deleted in the Sacy^tm1Lex^ locus, predicts a previously unappreciated promoter used for expression of sAC in mouse brain. Because sAC proteins in mouse brain derive from this alternate promoter, downstream from the deleted exons and inserted IRES-lacZ cassette, one would not expect to find LacZ expression in brain nor a neuronal defect in Sacy^tm1Lex^/Sacy^tm1Lex^ mice.

## Discussion

These findings reveal the sAC locus to be more complex than previously appreciated. The biochemically characterized sAC_t_ and sAC_fl_ isoforms may ultimately prove to be predominantly, if not exclusively, expressed in male germ cells, explaining the relatively specific male sterile phenotype of Sacy^tm1Lex^/Sacy^tm1Lex^ mice [11], [29]. In contrast, the presumptive promoter identified here, which directs expression of brain mRNAs initiating upstream of coding exon five, is likely to direct expression of sAC in many somatic tissues. Thus, the relatively subtle somatic phenotypes reported for Sacy^tm1Lex^/Sacy^tm1Lex^ mice [31] may be due to altered expression of a somatic sAC isoform instead of loss of sAC_t_ or sAC_fl_. Consistent with this hypothesis, we routinely required increased rounds of PCR amplification to detect sAC messages from Sacy^tm1Lex^/Sacy^tm1Lex^ tissues (Fig. 5).

Somatic isoforms encoded by transcripts from this promoter will possess only the second (C2) of the two identified catalytic domains [2]. Heterologous expression of C2-only containing isoforms has thus far failed to result in adenylyl cyclase activity [3], so how these isoforms produce cAMP remains an open question. By possessing only the C2 catalytic domain, somatic sAC isoforms will differ from the previously characterized, C1-C2 containing isoforms which may be exclusively expressed in male germ cells. Thus, it would be possible to design safe and effective contraceptive strategies by identifying inhibitors selective for C1-C2 containing sAC isoforms.

The evolutionary conservation of bicarbonate-mediated cAMP generation across many kingdoms [6], [36]–[39], including from the earliest known forms of life, Cyanobacteria [6], [36], suggests that this signal transduction pathway should be fundamentally important in biology. For example, multiple physiological processes, in addition to sperm function, are modulated by CO_2_ and/or HCO_3_^−^ (i.e., diuresis, breathing, blood flow, cerebrospinal fluid and aqueous humor formation) [40]. In most cases, the effects of CO_2_/HCO_3_^−^ have been ascribed to as yet undefined chemoreceptors [40]–[42], but potential links to cAMP signaling, such as in carotid body [43], suggest additional, somatic roles for a bicarbonate regulated adenylyl cyclase, such as sAC. With our identification of novel isoforms of sAC in somatic tissues, such additional roles remain possible.

## Materials and Methods

### Animals

2–4 month old wild type or Sacy^tm1Lex^/Sacy^tm1Lex^ mice [29] were euthanized with CO_2_, and brains, kidneys, or testis were immediately dissected, flash frozen in liquid N_2_ and stored at −80°C until processing. All animal work was performed with approval from the Institutional Animal Care and Use Committee of Weill Cornell Medical College (IACUC Protocol #0604-487A).

### Immunoprecipitation from detergent extracts

Brains or kidneys were thawed and homogenized in detergent lysis buffer in the presence of protease inhibitors (50 mM Tris, 150 mM NaCl, 0.4 mM EDTA, 0.1 mM DTT, 1 M PMSF, 10 μg/ml aprotinin, 10 μg/ml leupeptin, 1% NP40) (1∶10 w/v). All steps were performed on ice (or at 4°C) unless specified. Homogenates were centrifuged at 45,000xg for 50 minutes. The protein concentration of the supernatant fraction was determined (BioRad) and an aliquot saved at 4°C for Western analysis (‘pre-IP lysate’). Equivalent protein amounts from different supernatants were precleared by incubation with protein G beads (Amersham Pharmacia) (100 μl beads/100 mg total protein) overnight at 4°C. Samples were centrifuged at full speed in an Eppendorf centrifuge for 10′, and the supernatant was collected into fresh tubes. Clarified lysates were incubated with specific anti-sAC antibodies (R37 or R40) or control, mouse IgG at a concentration of 20 μg antibody/mg protein for 4 h at 4°C. Immune complexes were collected on Protein G beads (50 μl/100 mg total protein) and incubated for 1 h. Beads were collected by centrifugation, and an aliquot of the supernatant was collected for Western analysis (post-IP supernatant). Beads were washed three or four times in detergent-free lysis buffer.

For Western analysis, beads were incubated in SDS/PAGE sample buffer (BioRad) containing 5% β-mercaptoethanol for 5′ at room temperature, briefly spun, and an aliquot used for SDS/PAGE. Proteins were transferred to PVDF membranes, which were blocked in 5% milk (BioRad) for 1 hour at room temperature, rinsed once with TBST and incubated with biotinylated mAbs, R21 or R37 (1∶500 in TBST) overnight at 4°C. Control blots to examine streptavidin binding proteins were incubated in TBST alone. Membranes were rinsed in TBST (4×15′) and incubated with a HRP-conjugated streptavidin (1∶5000 in TBST) for 1 hour at room temperature. Bands were visualized using enhanced chemiluminescence (Pierce Co.)

For activity assays, beads were incubated in 100 μl reaction buffer containing 200 mM Tris pH 7.5, 100 U/ml phosphocreatine kinase, 20 mM creatine kinase, 2.5 mM ATP, and 10 mM MgCl_2_ for 30 minutes at 30°C. Where indicated, reactions contained 10 μM forskolin or 100 μM 4-hydroyestradiol (Steraloids, Inc.) or equivalent volumes of vehicle. Reactions were terminated by adding reaction supernatant into 100 μl 0.2 M HCl, samples were neutralized according to manufacturers protocol and cAMP quantitated using Correlate-EIA Direct Assay (Assay Designs, Inc).

**Antibody epitope mapping**

sAC_t_ sequence was first divided into 11 fragments, and primers were designed to amplify all 11 fragments, with forward primer 5′CACC overhang for cloning into pENTR/D-TOPO entry vector (Gateway System, Invitrogen) followed by ATG, where necessary. The entry clone was subsequently recombined with pDEST15 vector to create 11 sAC sequence fragments with N terminal GST tag. The N terminal tag was necessary to monitor protein expression and to increase fragment size to facilitate analysis by SDS-PAGE. Clones were shuttled into BL21-AI cells, and expression induced by addition of final concentration of 0.2% L-arabinose (Sigma) for 3–4 hours. Pelleted bacteria was resuspended in Laemmli sample buffer, run on SDS-PAGE and immunoblotted with each monoclonal antibody of interest. To narrow down the antibody epitope, forward and reverse complimentary primers encoding 14–17 amino acid stretches were designed to cover each of the recognized fragments. Each large fragment was covered by 5 overlapping smaller fragments. Forward primers contained CACC overhangs and N terminal ATG for cloning into pENTR/D-TOPO vector. Complimentary oligomers were annealed by incubation in cooling water in the presence of buffer containing 50 mM NaCl, 10 mM Tris-HCl pH 8, 10 mM MgCl_2_, 1 mM DTT, cloned into the entry vector, and recombined to generate GST-fusion proteins. Proteins were expressed and epitopes were defined by Western blotting using each monoclonal antibody.

### RNA production, and RT-PCR amplification of sAC products

Tissues harvested from wild type or Sacy^tm1Lex^/Sacy^tm1Lex^ mice were immediately placed in Trizol and either stored at −80°C or processed for total RNA according to manufacturer's protocol. Total RNA was quantified spectrophotometrically, and at least 2 mg of total RNA was used to generate polyA^+^ RNA using the Micro Poly(A) Purist Kit according to manufacturer's protocol (Ambion). Purified polyA^+^ RNA was resuspended in DEPC-treated water and treated with amplification grade DNase I according to the manufacturer's protocol (Invitrogen). DNase-free polyA^+^ RNA was stored at a final concentration of approximately 100 ng/mL at −80°C until use.

Approximately 500 ng of polyA^+^ RNA was used to generate first strand cDNA using Invitrogen's Platinum Taq PCR kit according to manufacturer's instructions. Briefly, RNA was incubated with 50 mM oligo(dT)_20_, (or 10 mM gene specific primer), 10mM dNTP and DEPC-treated water in a volume of 10 μl for 5 minutes at 65°C. An equal volume of cDNA Synthesis Buffer was added, yielding final concentrations of 1× Reverse Transcriptase Buffer (Invitrogen), 10 mM DTT, 125 mM MgCl_2_, 40U RNaseOUT, 200U SuperScript III Reverse Trancriptase, and the reaction was incubated for 60 minutes at 50°C. The reaction was terminated by incubation at 85°C for 5 minutes, and placed on ice. 1μl of RNase H (2 U/ml) was added, and incubated at 37°C for 20 minutes. This first strand was stored as single use aliquots at −80°C until use.

Routinely, PCR reactions used a standard three step protocol using Platinum Taq (Invitrogen, Inc.) with an initial denaturation step at 93°C for 3 minutes, followed by 35 or 40 cycles of 93°C for 20 seconds, 60°C for 20 seconds, and 68°C for 1 minute, followed by a final step at 68°C for 10 minutes. In wild type somatic tissues, 35 cycles was sufficient to detect sAC amplified products, but Sacy^tm1Lex^/Sacy^tm1Lex^ somatic tissues routinely required 40 rounds of amplification to detect fragments.

Primers used to amplify from exons 1 to 5:
Forward: LRL1127: 5′-ATGAGTGCGCGAAGGCAGGAAT-3′
Reverse: LRL1511: 5′-CTGCTCTCTGATCTGGAATCCTC-3′
Primers used in to amplify from new mRNA start site to exon 16:
Forward: Up5: 5′-ACCCAGAATGTGTTGTGCAAAC-3′
Reverse: LRL1519: 5′-CTTGTCCCGGATTTCCTGAGGCTG-3′
Primers used in to amplify from exons 15 to 16:
Forward: LRL1518: 5′-CAGAAGCAACTGGAAGCCCTG-3′
Reverse: LRL1519: 5′-CTTGTCCCGGATTTCCTGAGGCTG-3′
Primers used to amplify the βGal/Neo cassette:
Forward: LRL 1276: 5′-GGAACTAACAGAGATCTATCTGC-3′
Reverse: LRL 1277: 5′-GGATGGACCATCTAGAGACTGCCA-3′
Primers used to amplify β-actin:
Forward: BF: 5′-GGAGAAGATCTGGCACCACAC-3′
Reverse: BR: 5′-GGTGACCCGTCTCCGGAGTCC-3′
*5*′ *Rapid Amplification of cDNA Ends (5*′*RACE)*
5′RACE was performed on 500 ng of polyA^+^ RNA from brains of sACy^tm1Lex^/sACy^tm1Lex^ mice using 5′RACE Kit (Invitrogen) according to the manufacturer's protocol.
5′RACE Primers used from Exon 5:
Ex5GSP1: 5′-CTGCTCTCTGATCTGGAATCCTC-3′
Ex5GSP2: CAATTTCAATCATGCTCCGATCACAG
Ex5GSP3: CAGCAGTTTGGTGACAAAATAACGTCG
